# Circular RNA expression profiles following negative pressure wound therapy in burn wounds with experimental *Pseudomonas aeruginosa* infection

**DOI:** 10.1080/21655979.2021.2006965

**Published:** 2022-02-25

**Authors:** Yunshu Yang, Mengdong Liu, Fangfang Yang, Xujie Wang, Xiaozhi Bai, Shengzhi Mu, Yang Liu, Dahai Hu

**Affiliations:** a Department of Burns and Cutaneous Surgery, Xijing Hospital, Air Force Medical University, Xi’an, Shaanxi, China; b Key Laboratory of Resource Biology and Biotechnology in Western China, Ministry of Education, School of Life Sciences, Northwest University, Xi’an, Shaanxi, China; c Department of Burn and Plastic Surgery, Shaanxi Provincial People’s Hospital, Xi’an, Shaanxi, China

**Keywords:** Circular RNAs, negative pressure wound therapy, burn wound, *Pseudomonas aeruginosa*, whole-transcriptome sequencing

## Abstract

Infections of burn wounds, especially those caused by *Pseudomonas aeruginosa*, could trigger sepsis or septic shock, which is the main cause of death after burn injury. Compared with traditional saline-wet-to-dry dressings, negative pressure wound therapy (NPWT) is more effective for the prevention and treatment of wound infections. However, the mechanism by which NPWT controls infection and accelerates wound healing remains unclear. Accordingly, in this study, the molecular mechanisms underlying the effects of NPWT were explored using a murine model of *P. aeruginosa*-infected burn wounds. NPWT significantly reduced *P. aeruginosa* levels in wounds, enhanced blood flow, and promoted wound healing. Additionally, NPWT markedly alleviated wound inflammation and increased the expression of wound healing–related molecules. Recent evidence points to a role of circular RNAs (circRNAs) in wound healing; hence, whole-transcriptome sequencing of wound tissues from NPWT and control groups was performed to evaluate circRNA expression profiles. In total, 12 up-regulated and 25 down-regulated circRNAs were identified between groups. Among these, five significant differentially expressed circRNAs acting as microRNA sponges were identified, and their predicted targets were verified by reverse transcription-quantitative polymerase chain reaction. These results further support the roles of circRNAs in wound healing by NPWT and the prevention of *P. aeruginosa* infection, providing key molecular targets for further functional analyses.

## 1. Introduction

As one of the most lethiferous complications of severe burns, burn wound infection is associated with a high rate of mortality owing to the development of sepsis or septic shock [1,2]. In recent years, multidrug-resistant bacteria have become the leading cause of death, and *Pseudomonas aeruginosa* is the most common etiological agent of serious infection in burn patients [3–5]. Although traditional saline-wet-to-dry dressings could drain wound secretions [6], they are not sufficient to completely remove *P. aeruginosa* [7]. Hence, preventing and treating burn wounds infected with drug-resistant *P. aeruginosa* remain important clinical challenges [1,3–5].

Negative pressure wound therapy (NPWT) is a widely-used management for burn and trauma, which has proven to be highly effective for wound infections [8,9]. NPWT can improve the wound environment by draining excessive effusion, alleviating interstitial edema, and reducing the capillary afterload in local tissues [9,10]. The airtight negative pressure environment generated by NPWT effectively isolates wounds from the external environment, thus destroying hotbeds of bacterial growth and cross-infection. Additionally, the relatively anoxic atmosphere created by NPWT can suppress bacterial growth and promote the proliferation of fibroblasts, thereby significantly accelerating wound healing [11]. Moreover, NPWT was reported to cause a remarkable and sustained decrease of *P. aeruginosa* levels in wounds [12]. Despite implications for its clinical usage, the specific molecular mechanisms underlying these beneficial effects of NPWT remain uncertain.

With advances in next-generation sequencing, RNA-sequencing has become the fastest and most effective approach to find connections between molecular mechanisms and disease phenotypes [13,14]. To date, RNA-sequencing has provided support for the important roles of non-coding RNAs (ncRNAs) in multiple biological processes [15]. Competitive endogenous RNAs (ceRNAs) are ncRNAs [including long non-coding RNAs, pseudogene transcripts, and circular RNAs (circRNAs)] that compete for the same microRNA (miRNA) targets and thereby participate in post-transcriptional regulation [16,17]. Studies have shown that ceRNAs, particularly circRNAs, play essential regulatory roles in skin wound healing [18,19]. However, no study has assessed whether circRNAs are involved in the mechanism by which NPWT can protect against burn wound infection and sepsis.

Therefore, in this study, we investigated the effects of NPWT on burn wound healing and related sepsis in a *P. aeruginosa* infection burn mouse model. We further identified the circRNAs profile and related ceRNA networks following NPWT in the burn wound infection model via a high-throughput RNA-sequencing approach.

## 2. Materials and methods

### 2.1. Bacterial strain and culture conditions

To establish fluorescently labeled *P. aeruginosa*, the *Photorhabdus luminescens* luxCDABE operon was introduced to the wild-type *P. aeruginosa* PAO1 parental strain (#47,085; American Type Culture Collection, Manassas, VA, USA). After the bacteria were plated, a monoclonal colony was selected and amplified in Luria–Bertani liquid medium overnight at 37°C until the optical density reached 0.8 at 600 nm.

### 2.2. Mouse model of burn wound sepsis

Eight- to twelve-week-old specific pathogen-free male C57B6/L mice were purchased from the Experimental Animal Center of the Air Force Medical University (Xi’ an, Shaanxi, China). All procedures were carried out in accordance with the ARRIVE guidelines and were approved by the Ethics Committee of Air Force Medical University (No. XJYYLL-2017133). A total of 120 mice were randomly and equally divided into two groups: the ‘Scald + Infection’ and ‘Sham + Infection’ groups. In the ‘Scald + Infection’ group, a third-degree scald of 2 cm diameter was generated on the shaved back of each mouse using water vapor by continuous scalding for 4 s; the wound occupied approximately 6–8% of the body surface area. Subsequently, 50 μl of fluorescently labeled *P. aeruginosa* (1.0 × 10^6^ colony-forming units/ml) was inoculated onto the eschar. When the bacteria solution was completely absorbed, the mice were allowed to recover. In the ‘Sham + Infection’ group, normal saline was smeared onto the skin surface but without the scalding step. Six mice were randomly selected from each group for evaluation on days 1, 3, 5, and 7 post-infection (*P. aeruginosa* inoculation) and then sacrificed to collect tissue samples. Survival was observed every 24 h for 7 days (n = 12) (Figure 1a).

**Figure 1.** **Construction of a murine model of burn wound sepsis involving *P. aeruginosa* infection**. (a) Schematic diagram of the procedure, including scald, bacterial inoculation, escharectomy, and NPWT following model establishment. (b) *P. aeruginosa* count after scald or sham treatment analyzed by bacterial culture and colony computation on days 1, 3, 5, and 7 after model establishment. (c) Survival rates of mice without *P. aeruginosa* infection after scald or sham treatment. (d) Enzyme-linked immunosorbent assays to measure IL-1β and IL-6 levels in the serum from mice on days 1, 3, 5, and 7 after model establishment. (e) Fluorescence intensity of wound bacteria on days 1, 3, 5, and 7 after model establishment. *P < 0.05 and ****P < 0.0001. Abbreviation: NPWT, negative pressure wound therapy.

### 2.3. NPWT

Ninety mice were modeled as described above for the ‘Scald+ Infection’ group and then randomly splitted into the NPWT and negative control groups. In both groups, the wounds were covered with polyurethane foam and blocked with a biologic semi-permeable membrane. In the NPWT group, the wounds were subjected to NPWT with continuous negative pressure suction of – 120 mmHg. In the control group, the wounds were cleaned with a sterile saline solution, and the dressing was changed once every 24 h. Tissue samples were collected and evaluated on days 1, 3, 5, and 7 (Figure 1a).

### 2.4. P. aeruginosa *counts*

After cleaning the surface exudates with sterile saline solution, tissue biopsies were collected from three different points of the wound from each mouse under gnotobiosis on days 1, 3, 5, and 7. Tissues were ground and mixed with an equivalent amount of 0.9% saline. Each sample of homogenate at a final dilution of 1:1,000 was inoculated onto Luria-Bertani medium on (agar) plates and cultured for 24 h to determine the *P. aeruginosa* counts per gram of tissue. The biopsies were processed and evaluated blindly by a medical microbiologist.

### 2.5. In vivo *fluorescence imaging*

Images of wounds were obtained on days 0, 1, 3, 5, and 7 after model establishment. After the mice were euthanized, the IVIS 2000 system was used to capture bioluminescent *P. aeruginosa* on the wounds with a 1-min exposure. Binning of four images was used to increase sensitivity without compromising the spatial resolution. Images were quantitatively analyzed using Living Image, version 3.0 (Xenogen, Alameda, CA, USA).

### 2.6. Wound blood flow imaging

Blood flow in the wounds and the area around wounds was detected using a laser Doppler flowmeter (#PeriFlux 5000; Perimed AB, Stockholm, Sweden). An ultrasound probe was fixed at a distance of 16 cm from the wound, and the average perfusion range was defined as the diagonal intersection of the square with a median side of 5 cm sharing the center of the wound. The results are presented in perfusion units.

### 2.7. Wound healing observation

Images of wounds were obtained on days 0, 1, 3, 5, and 7 after NPWT. The healing rates were calculated by the gray values of the wound healing area normalized against the quantitative value for day 0.

### 2.8. Enzyme-linked immunosorbent assay (ELISA)

Mouse blood samples were collected retro-orbitally and centrifuged at 3,000 rpm for 20 min. The upper layer of the serum was then assayed using ELISA kits to measure the levels of interleukin (IL)-1β (Bosterbio, #EK0394) and IL-6 (Bosterbio, #EK0411).

### 2.9. Hematoxylin–eosin (H&E) staining

Mouse wound tissue samples were fixed in 4% paraformaldehyde, embedded in paraffin, and cut into 5-μm-thick sections. The sections were stained with H&E, and images were obtained under an FSX100 microscope (Olympus, Tokyo, Japan). Five high-magnification images were randomly selected for analyses.

### 2.10. Immunohistochemical staining

Immunohistochemical staining was performed using representative tissue samples fixed in 4% paraformaldehyde, embedded in paraffin, and cut into 5-μm-thick sections. After antigen recovery and blocking in goat serum, the tissue sections were incubated with primary antibodies against CD31 (#ab9498; Abcam, Cambridge, UK), Ki67 (#ab15580; Abcam), vascular endothelial growth factor (VEGF; #sc-20,718; Santa Cruz Biotechnology, Santa Cruz, CA, USA), and transforming growth factor (TGF)-β1 (#sc-6319; Santa Cruz) overnight and visualized using the HRP-DAB Kit (#CTS005; R&D Systems, Minneapolis, MN, USA) the next day. The staining was quantified by calculating the average of positive staining cells of 5 random sights (200×).

### 2.11. RNA-sequencing

Total RNA was extracted using TRIzol reagent (#9109; Takara, Kusatsu, Japan) and purified using Dynabeads™ Oligo(dT)25 (#61,002; Invitrogen, Carlsbad, CA, USA). A cDNA library for sequencing was constructed following the instructions provided with the NEB kit (#7530; New England Biolabs, Ipswich, MA, USA). High-throughput sequencing using the Illumina HiSeq Xten system and relevant bioinformatics analyses were performed by Shanghai Novelbio Ltd. (Shanghai, China). The expression levels of genes in each sample were normalized to units of fragments per kilobase of transcript per million mapped reads. The DEseq algorithm was applied to filter the differentially expressed genes (DEGs) according to a false discovery rate-adjusted *P*-value of <0.05 and fold change (FC) >2 or <0.5. Gene Ontology (GO) terms and pathway enrichment of DEGs were identified using the AmiGO database and Kyoto Encyclopedia of Genes and Genomes (KEGG) database, respectively.

### 2.12. Reverse transcription-quantitative polymerase chain reaction (RT-qPCR)

Total RNA was extracted using TRIzol reagent (#9109; Takara). In total, 1000 ng of isolated RNA was reverse-transcribed into cDNA using Prime Script™ RT Reagent Kit (#RR036A-1; Takara). qPCR was then performed using CFX Connect Real-time System (BIO-RAD, Hercules, CA, USA) with SYBR Premix Ex Taq™ (Takara, #RR420A) and specific primers. Relative expression levels were calculated by the 2^−ΔΔCt^ method with normalization against the *Gapdh* expression level. MiRNAs cDNA was synthesized using a miR-X miRNA First-Strand Synthesis Kit (Takara, #638315). Polyadenylation reverse transcription were performed at 37°C for 10 sec and 60°C for 30 sec. Quantification of miRNA by qPCR was executed using SYBR Advantage qPCR Premix (Takara, #639676) with an initial denaturation step at 95°C for 10 sec, followed by 42 cycles at 95°C for 5 sec and 60°C for 20 sec. U6 snRNA was used as the internal control to normalize the expression. The primer sequences for each gene are listed in Table 1.

**Table 1.** The primer sequences for each gene

**Gene**	**Forward**	**Reverse**
Il10ra	TTGTCGCGTTTGCTCCCATT	GAAGGGCTTGGCAGTTCTG
Inpp5d	GAGACACTGTTTCAGCGTCTAC	CGTCTTCAAAAAGTCGGAATCCA
Prkcb	ATGAGTTCGTCACGTTCTCCT	CCATACAGCAGCGATCCACAG
Plcb2	TGCTGATCGAAAACGGGTGG	AGCTTTAGAGTGGTAGGAAGTGA
Eif2ak2	ATGCACGGAGTAGCCATTACG	TGACAATCCACCTTGTTTTCGT
Lamc3	CAGAAAACCTATGGCCGTCCT	CCAAACGTGTTGAGCCGATCT
Adcy1	GTCACCTTCGTGTCCTATGCC	TTCACACCAAAGAAGAGCAGG
Wnt7b	CTTCACCTATGCCATCACGG	TGGTTGTAGTAGCCTTGCTTCT
mmu_circ_0001240	TACCAGATTCCCAGGCTCCAA	CATTCACACTGGCTAATGCAGG
mmu_circ_0011322	TGATGCAGGACAGTACCGCT	CCTGATGATGCTTCCGCTTTG
mmu_circ_0004796	GCAGATGTCCCTTTGGCTGA	GCTCATGCATCATGGTCCTTT
mmu_circ_0013121	CGTCAGACTGCTTTCTCACTGT	CTTTCTGCCCTCACTCCAACA
mmu-miR-497a-5p	CAGCAGCACACTGTGGTTTGTA	
mmu-miR-1224-3p	CCCCACCTCTTCTCTCCTCAG	
mmu-miR-669m-5p	TGTGTGCATGTGCATGTGTGTAT	
mmu-miR-877-3p	TGTCCTCTTCTCCCTCCTCCC	

### 2.13. Statistical analysis

All quantitative results were presented as mean ± SD. Survival was analyzed by the Kaplan-Meier and log-rank t-test. The differences between the mean variables of the two groups were determined using Student’s t test. Analysis of variance (ANOVA) with Tukey’s post hoc test was used for multiple group analyses. Statistically significant differences were considered at *P* < 0.05. For all statistical tests, *P < 0.05, **P < 0.01, ***P < 0.001, ****P < 0.0001 and ns mean no significance. Statistical analysis was conducted with GraphPad Prism 8.0 software.

## 3. Results

### 3.1. Study design

To better understand the beneficial effects of NPWT on wound healing, we engineered the *P. aeruginosa* parental PAO1 strain using an operon carrying a fluorescence reporter gene and then constructed a murine model of burn wounds with *P. aeruginosa* infection. Bioluminescent imaging, *P. aeruginosa* counts, and proinflammatory cytokine detection were performed to monitor the infection condition and inflammation of the local wounds. Laser Doppler perfusion imaging, wound healing rate calculation, and staining of wound healing–related molecules were performed to assess wound healing conditions. To further search for the underlying circRNAs involved in infectious wound healing after NPWT, a high-throughput RNA-sequencing approach was conducted, and subsequent ceRNA network analyses were performed to understand the biological functions of identified circRNAs and their target genes.

### 3.2. *Successful establishment of a murine model of burn wound sepsis involving* P. aeruginosa *infection*

To assess the ability of NPWT to control wound sepsis, we first constructed a murine model of a third-degree scald wound or sham wound, which was experimentally infected with *P. aeruginosa*. Levels of *P. aeruginosa* were monitored on days 1, 3, 5, and 7, and survival rates were observed over 7 days. *P. aeruginosa* counts in the ‘Scald + Infection’ group were dramatically higher than those in the ‘Sham + Infection’ group on days 3, 5, and 7 (Figure 1b). Consistent with these findings, analyses of fluorescence intensity, as determined by *in vivo* bioluminescent imaging, showed that the bacteria count in the wounds after scalding was markedly higher in the ‘Scald + Infection’ group than in the ‘Sham + Infection’ group, and the intensity peaked on day 3 in both groups (Figure 1e). Moreover, the ‘Scald + Infection’ group had a significantly higher mortality rate than the ‘Sham + Infection’ group (Figure 1c). Additionally, ELISA showed that the levels of secreted pro-inflammatory cytokines IL-1β and IL-6 were significantly increased in the mice of the ‘Scald + Infection’ group compared with those of the ‘Sham + Infection’ group (Figure 1d). Together, these results indicated that the murine model of burn wound sepsis with *P. aeruginosa* infection was successfully established.

### 3.3. *NPWT significantly reduced* P. aeruginosa *in wounds, promoted wound healing, and alleviated sepsis-related organ injuries*

To clarify the effects of NPWT on burn wound infection, mice with or without NPWT following burn wound sepsis were evaluated by *in vivo* bioluminescent imaging. Compared with that in the control group, the fluorescence in the NPWT group was less intense and showed a decreasing trend over time (Figure 2a). The culture results also indicated that NPWT markedly reduced *P. aeruginosa* counts in the wounds (Figure 2c). In both assays, the difference between groups was more significant on day 3 than at any other evaluation time point (Figures 2a & 2c).

**Figure 2.** **NPWT significantly reduced *P. aeruginosa* counts in wounds, promoted wound healing, and alleviated sepsis-related organ injuries**. (a) Fluorescence intensity of wound bacteria detected on days 1, 3, 5, and 7 with or without NPWT (n = 6). (b) Laser Doppler perfusion imaging for the detection of wound blood perfusion (n = 6). (c) *P. aeruginosa* were counted by culture and colony computation (n = 6). (d) Wound healing rates were calculated based on the gray values of wound healing areas (n = 15). (e) Survival rates of mice with NPWT or control treatment. (f) Hematoxylin-eosin staining of mouse skin, liver, lung, and kidney tissue samples from the NPWT and control groups (n = 6; scale bar = 50 μm). *P < 0.05, **P < 0.01, ***P < 0.001, ****P < 0.0001. Abbreviation: NPWT, negative pressure wound therapy.

Doppler ultrasound showed that NPWT conspicuously increased the wound blood flow (Figure 2b) and significantly increased the wound healing rate on days 3, 5, and 7 posttreatment (Figure 2d). These findings suggested that NPWT had a protective effect against *P. aeruginosa* in wounds and promoted wound healing.

Further to determine whether NPWT is effective for improving general conditions, the survival rate after treatment with NPWT or saline wet dry dressing was monitored for 72 h. We found that NPWT dramatically reduced the mortality of mice with burn wound sepsis (Figure 2e). Consistently, H&E staining of the mouse skin, lung, liver, and kidney tissue samples revealed that NPWT ameliorated organ injuries, as evidenced by alleviated cell edema and hemorrhage, reduced inflammatory exudation, and relatively intact structural integrity (figure 2f). Collectively, these findings demonstrated that NPWT not only alleviated the local infection and inflammation of burn wounds, thereby promoting wound healing, but also relieved systemic sepsis and organ injuries.

### 3.4. NPWT alleviated wound inflammation and increased the expression of wound healing–related molecules

To further verify the role of NPWT in controlling the inflammatory response to wound infection, RT-qPCR was utilized to evaluate the mRNA levels of pro-inflammatory cytokines, including *Il1β, Il6, Il12*, and tumor necrosis factor-alpha (*Tnfa*). NPWT remarkably decreased the levels of all four inflammatory cytokines, and the difference increased over time but peaked at different time points, either on day 3 or day 5 (Figure 3a).

**Figure 3.** **NPWT alleviated wound inflammation and increased the expression of wound healing–related molecules**. (a) Inflammatory cytokines, including IL-1β, IL-6, IL-12, and TNF-α, in wounds on days 0, 1, 2, 3, 5, and 7 analyzed by RT-qPCR. (b) *Vegf* and *Tgfβ1* mRNA levels analyzed by RT-qPCR. (c) H&E staining of wound tissues on day 3 in the NPWT group and control group (n = 6). (d) Immunohistochemical staining for CD31, Ki67, TGF-β1, and VEGF in wound tissues on day 3 in the NPWT group and control group (n = 6). *P < 0.05, ****P < 0.0001. Abbreviations: NPWT, negative pressure wound therapy; H&E, hematoxylin and eosin; RT-qPCR, reverse transcription-polymerase chain reaction.

Based on our observations that infection control and wound healing by NPWT were most notable on day 3 after treatment, we focused on this time point for further analyses of mouse tissues. H&E staining revealed that NPWT obviously promoted wound tissue repair, as evidenced by reduced inflammatory exudates and the relatively intact structural integrity of the skin. Immunohistochemistry staining was used to evaluate markers of wound-healing conditions, including CD31 for wound angiogenesis, Ki67 for cell proliferation, TGF-β1 for tissue repair, and VEGF for the new capillary density. These four wound healing–related molecules were highly expressed in mouse tissues from the NPWT group compared to the control group. Taken together, these results indicated that NPWT strikingly alleviated wound inflammation and increased the expression of wound healing–related molecules.

### 3.5. Clustering analysis of DEGs and circRNAs between the NPWT and control groups

We conducted whole-transcriptome sequencing of wound tissues in the NPWT and control groups for a comparative analysis of samples obtained on day 3. A total of 864 significant differentially expressed mRNAs were identified, including 610 up-regulated and 254 down-regulated genes in the NPWT group (Figure 4a). Additionally, 37 significantly differentially expressed circRNAs were identified, including 12 up-regulated and 25 down-regulated loci in the NWPT group, as shown by hierarchical clustering analysis (Figure 4b). Among these circRNAs, 29 were located in protein-coding exons and were selected for further analyses of regulatory networks.

**Figure 4.** **Heatmap of the clustering analysis of differentially expressed** (a) **mRNAs and** (b) **circRNAs between the NPWT and control groups**. Down-regulated and up-regulated molecules in the NPWT group are shown in green and red, respectively. Abbreviations: circRNA, circular RNA; NPWT, negative pressure wound therapy.

### 3.6. Integrated analysis of circRNA–miRNA–mRNA networks

Focusing on the 29 exonic circRNAs, MiRanda and NovelBio were used for integrated analysis of circRNA–miRNA–mRNA networks. Five circRNAs with five predicted miRNA-binding sites and ceRNA-regulatory relationships were identified and annotated according to sequence-pairing predictions (Figures 5a & 5b). Among these, the expression levels of chr13_76759820_76741294_+18,526-Mctp1 (mmu_circ_0004796) and chr4_137557440_137557174_+266-Hspg2 (mmu_circ_0011322) were increased following NWPT with log_2_FC values of 3.66 and 20, respectively. The levels of chr4_108719812_1087177 89_-2023-Zfyve9 (mmu_circ_0001240), chr6_13476 1434_134758619_-2815-Dusp16 (mmu_circ_0013121), and chr17_80053641_80044494_-9147-Hnrnpll (circRNA Hnrnpll) were down-regulated following NWPT, with log_2_FC values of – 2.33, – 1.74, and – 1.32, respectively. Based on associations between the expression levels of these five circRNAs and miRNAs, various miRNAs, including mmu-miR-877-3p, mmu-miR-669 m-5p, mmu-miR-1224-3p, and mmu-miR-497a-5p, were predicted to have ceRNA-regulatory relationships. Additionally, 52 target mRNAs were identified, forming circRNA–miRNA–mRNA networks (Figure 5a). The predicted combinations were based on the detection of complementary sequences in circRNAs and corresponding miRNAs (Figure 5b).

**Figure 5.** **Integrated analysis of circRNA–miRNA–mRNA networks**. (a) Prediction of circRNAs involved in circRNA–miRNA–mRNA interaction networks. (b) Combination of circRNAs and miRNAs. Abbreviations: circRNA, circular RNA; miRNA, microRNA.

Furthermore, we evaluated the functions of all significant DEGs in circRNA–miRNA–mRNA regulatory relationships based on GO and KEGG pathway analyses. The top 15 enriched GO analysis terms in the biological process, molecular function, and cellular component categories included innate immune response, inflammatory response, Toll-like receptor signaling pathway, MyD88-dependent Toll-like receptor signaling pathway, iron ion homeostasis, intracellular signal transduction, defense response to virus, defense response to protozoan, pigment granule organization, defense response to fungus, defense response to gram-negative bacterium, regulation of cytokine secretion, defense response to gram-positive bacterium, and chemotaxis (Figure 6a). A KEGG pathway integrated analysis of circRNAs–miRNAs–mRNAs revealed enrichment in the chemokine signaling pathway, leukocyte trans-endothelial migration, neuroactive ligand-receptor interaction, cytokine-cytokine receptor interaction, Rap1 signaling pathway, Chagas disease (American trypanosomiasis), B cell receptor signaling pathway, cholinergic synapse, oxytocin signaling pathway, amoebiasis, focal adhesion, Fc gamma R-mediated phagocytosis, NF-kappa B signaling pathway, melanogenesis and African trypanosomiasis (Figure 6b).

**Figure 6.** **GO and KEGG pathway analyses of circRNA targets**. (a) GO analysis of target genes in circRNA–miRNA–mRNA networks. (b) KEGG pathway analysis of target genes in circRNA–miRNA–mRNA networks. Abbreviations: circRNA, circular RNA; miRNA, microRNA; GO, Gene Ontology; KEGG: Kyoto Encyclopedia of Genes and Genomes.

### 3.7. Verification of DEG expression profiles

To verify the RNA-sequencing results, RT-qPCR was used to evaluate the expression of five circRNAs and four miRNAs with a predicted ceRNA-regulatory relationship. In accordance with the prediction results, the circRNAs chr4_108719812_108717789_-2023-Zfyve9 (mmu_circ_0001240), chr6_134761434_134758619_-2815-Dusp16 (mmu_circ_0013121), and chr17_80053641_80044494_-9147-Hnrnpll (circRNA Hnrnpll), and the miRNAs mmu-miR-497a-5p and mmu-miR-1224-3p exhibited varying degrees of declined expression after NWPT (Figures 7a & 7b). Additionally, RT-qPCR results confirmed the up-regulation of chr13_76759820_76741294_+18,526-Mctp1(mmu_circ_0004796), chr4_137557440_137557174_+266-Hspg2 (mmu_circ_0011322), and mmu-miR-877-3p, and mmu-miR-669 m-5p in the NPWT group (Figures 7a & 7b). Furthermore, among the 52 predicted mRNA targets, we selected eight for validation, namely, *Il10ra, Inpp5d, Prkcb, Plcb2, Eif2ak2, Lamc3, Adcy1*, and *Wnt7b*, based on their significant involvement in infection-related pathways in the KEGG analysis (Figure 6b); the mRNA levels of these DEGs are presented in Figure 7c.

**Figure 7.** **Transcriptional verification of differential expression profiles**. Relative expression levels of five circRNAs (a), four miRNAs (b), and selected mRNAs (c) in predicted ceRNA-sponge networks detected by RT-qPCR in the NPWT and control groups. The data are presented as means ± standard errors of the mean of at least three independent experiments. Abbreviations: circRNA, circular RNA; NPWT, negative pressure wound therapy; miRNA, microRNA; RT-qPCR, reverse transcription-quantitative polymerase chain reaction.

## 4. Discussion

Burn wounds are a major route for pathogen invasion. Without effective wound management, the invasive infection may expand and result in wound sepsis, which is characterized by rapid deterioration and high fatality rates [20,21]. Moreover, deep burn wounds act as breeding grounds for bacterial infections, involving multiple pathological processes such as the local disturbance of blood circulation, tissue edema, and inflammatory response, resulting in non-healing wounds [22].

Since the development of NPWT in 1993 by Fleischman et al. [23], its clinical use has increased substantially, demonstrating superior efficacy over other approaches. However, the molecular mechanisms by which NPWT effectively controls wound infection and promotes wound healing have not been elucidated to date. Hence, in this study, we established a *P. aeruginosa* infection model following a third-degree burn on the backs of mice to evaluate the therapeutic and biological effects of NPWT. By whole-transcriptome sequencing, we further investigated the molecular changes induced by NPWT in the treatment of severe infected complex burn wounds.

Basic research and multiple clinical reports have confirmed the efficacy and utility of NPWT in improving wound conditions and promoting wound healing, revealing that NPWT could effectively control local infection and excessive inflammation [12,24,25]. Lallis et al. [12] found that *Pseudomonas* levels in wounds could be decreased to a substantially greater extent by NPWT than by traditional saline-wet-to-dry dressings. Additionally, in a rabbit ear biofilm infection model, NPWT weakened the motility of *P. aeruginosa*, thus enhancing wound healing [24]. Our study confirmed these beneficial effects of NPWT in clearing *P. aeruginosa* from wounds, as determined by fluorescence imaging of luminous *P. aeruginosa* and bacterial culture counts. In our model, NPWT had the most significant effects from days 3 to 7, suggesting that this approach has a continuous influence on *P. aeruginosa* proliferation. Furthermore, it is widely accepted that the inflammation accompanying infection is a principal factor affecting wound healing [26]. In support of this, our analysis of pro-inflammatory cytokines, including IL-1β, IL-6, IL-12, and TNF-α, confirmed that NPWT could alleviate the local inflammatory response in wounds induced by *P. aeruginosa* infection.

In addition, NPWT has been shown to accelerate wound healing by improving local perfusion and promoting angiogenesis [10,27,28]. Indeed, we also found that NPWT dramatically elevated the levels of TGF-β1 and VEGF, indicating that it promotes granulation tissue proliferation and new blood vessel generation. Immunohistochemical staining of CD31 and Ki67 additionally revealed the therapeutic effect of NPWT in facilitating wound healing by promoting angiogenesis and cell proliferation.

CircRNAs, as a newly defined subset of ncRNAs, exert important biological effects by acting as miRNA or protein inhibitors (so-called ‘sponges’) via regulating protein function or being translated themselves [29]. Accordingly, circRNAs are important for the regulation of numerous physiological or pathological processes, including wound repair. Yang et al. [30] found that the circRNA circ-Amotl1 accelerates the wound healing process in NIH3T3 fibroblasts and in a mouse excisional wound model via interaction with STAT3, further modulating DNMT3a and miR-17-5p expression. Nuutila et al. [31] provided initial insight into the molecular mechanisms underlying the effects of NPWT on wound closure and healing on split-thickness skin graft donor sites by genome-wide microarrays; however, circRNA expression profiling of NPWT in wound healing was not performed. Applying a whole-transcriptome sequencing approach, we further screened differentially expressed circRNAs in *P. aeruginosa*-infected wounds after NPWT. We identified 12 up-regulated and 25 down-regulated circRNAs in mice that received NPWT compared with those that received control dressings on the *P. aeruginosa*-infected wounds. In particular, five significant differentially expressed circRNAs showed miRNA-sponge regulatory relationships, including chr13_76759820_76741294_+18,526-Mctp1(mmu_circ_0004796), chr4_137557440_137557174_+266-Hspg2 (mmu_circ_0011322), chr4_108719812_108717789_-2023-Zfyve9 (mmu_circ_0001240), chr6_134761434_134758619_-2815-Dusp16 (mmu_circ_0013121), and chr17_80053641_80044494_-9147-Hnrnpll (circRNA Hnrnpll); none of these circRNAs has been identified to play a role in the wound-healing process to date.

Although the target miRNAs of the differentially expressed circRNAs identified in this study, including mmu-miR-877-3p, mmu-miR-669 m-5p, mmu-miR-1224-3p, and mmu-miR-497a-5p, have also not been linked to wound healing previously, miR-877-3p and miR-1224-3p have been reported to be associated with cell proliferation and migration in tumors [32,33]. Additionally, miR-497a-5p and miR-1224-3p appear to contribute to inflammatory responses [34,35].

We further evaluated the roles of these five circRNAs in the regulation of physiological or pathological processes by GO and KEGG pathway analyses. The enriched KEGG pathways, including the chemokine signaling pathway, leukocyte trans-endothelial migration, cytokine-cytokine receptor interaction, and NF-kappa B signaling pathway, indicated that these circRNAs are closely related to immune and inflammatory responses.

Genes identified in the predicted circRNA–miRNA–mRNA networks were validated by RT-qPCR. The results for the five circRNAs, four miRNAs, and target mRNAs were generally consistent with the sequencing and prediction results. In particular, the levels of the five circRNAs and the two predicted miRNA targets mmu-miR-877-3p and mmu-miR-669 m-5p were significantly increased, and the levels of mmu-miR-1224-3p and mmu-miR-497a-5p were significantly decreased by NPWT.

Collectively, this study demonstrates the successful establishment of a novel *P. aeruginosa* infected burn wound model and reveals the protective role of NPWT in wound healing and systemic sepsis. Moreover, we identified the circRNA expression profile of the effects of NPWT in infected burn wounds, identifying five circRNAs (mmu_circ_0004796, mmu_circ_0011322, mmu_circ_0001240, mmu_circ_0013121, and circRNA Hnrnpll), which act as miRNA sponges, and the related miRNAs were identified as mmu-miR-877-3p, mmu-miR-669 m-5p, mmu-miR-1224-3p, and mmu-miR-497a-5p. Overall, our discovery yields several novel ncRNA targets of NPWT in burn wound sepsis, which can further offer potential new therapeutic targets. Despite this advance in our understanding of circRNAs in NPWT, further experiments are required to substantiate whether the ceRNA networks identified ultimately play a role in burn wound sepsis.

## Conclusions

This study demonstrates that NPWT could significantly accelerate wound healing by reducing the *P. aeruginosa* quantity, alleviating wound inflammation, and promoting angiogenesis in a *P. aeruginosa* infected burn wound model. NPWT also significantly ameliorated systemic inflammation and related organ injuries to prevent burn wound sepsis. We identified the circRNA profiles related to the effect of NPWT on the infected burn wound, and five significant circRNAs acting as miRNA sponges and the related miRNAs were identified. Further exploration of the role of the predicted circRNA-miRNA-mRNA networks is required to elucidate the deeper mechanism of NPWT in burn wound sepsis. The identified circRNAs offer promising targets for wound and sepsis therapy.

## Data Availability

All data and materials generated or used during the study appear in the submitted article.

## List of abbreviations

NPWT: negative pressure wound therapy

ncRNA: non-coding RNA

ceRNA: competitive endogenous RNA

circRNA: circular RNA

miRNA: microRNA

IL: interleukin

H&E: hematoxylin and eosin

VEGF: vascular endothelial growth factor

TGF: transforming growth factor

DEG: differentially expressed gene

FC: fold change

GO: Gene Ontology

KEGG: Kyoto Encyclopedia of Genes and Genomes

RT-qPCR: reverse transcription-quantitative polymerase chain reaction
